# Molecular Pathways Involved in Promoting Activity of Timosaponin BII on Hair Growth in C57BL/6 Mice

**DOI:** 10.1155/2020/9451596

**Published:** 2020-09-18

**Authors:** Lei Xiao, Xia Zhang, Zhiyi Chen, Jianhua Li, Bing Li, Lin Li

**Affiliations:** ^1^School of Food Science and Engineering, Guangdong Province Key Laboratory for Green Processing of Natural Products and Product Safety, South China University of Technology, Guangzhou 510640, China; ^2^Infinitus (China) Co., China; ^3^Sericultural & Agri-Food Research Institute, Guangdong Academy of Agricultural Sciences, Key Laboratory of Functional Foods, Ministry of Agriculture and Rural Affairs, Guangdong Key Laboratory of Agricultural Products Processing, Guangzhou 510610, China; ^4^School of Chemical Engineering and Energy Technology, Dongguan University of Technology, College Road 1, Dongguan 523808, China

## Abstract

Hair loss is a common disease in dermatology, while the approved drugs may have unpredictable side effects. In this study, the effect of timosaponin BII extracted from *Anemarrhena asphodeloides* on hair growth of C57BL/6 mice was investigated by measuring the hair follicle morphology, hair growth length and area in C57BL/6 male mice, and the immunohistochemical analysis of *β*-catenin, Wnt3a, and Wnt10b in the dorsal skins of mice after topical application with minoxidil and timosaponin BII for 15 days. The decrease in skin brightness, the increase in the regrowing area of hair and hair follicles numbers, and the improvement of hair follicle morphology in the group applied with 0.5% timosaponin BII indicated an induction of the anagen phase in telogenic mice skin, which were comparative to the 2% minoxidil treatment. The immunohistochemical analysis detected an increase in the expression of *β*-catenin and Wnt10b, supporting the theory of the activation of the *β*-catenin/Wnt pathway was one of the pathways that are related to anagen phase induction. *Anemarrhena asphodeloides* is a herb commonly used for metabolic disorders in China. The present study is the first to show that the timosaponin BII, which is present at a high concentration in *A. asphodeloides*, promotes hair growth in C57BL/6 male mice. The results indicate that timosaponin BII may be a potential promoting agent for hair growth.

## 1. Introduction

Hair loss or alopecia is one of the common diseases in dermatology; although it is not a life-threatening illness it can bring great painful suffering on human mental stress over a lifetime. The rate of adult male hair loss is 25% and that of females is 22% in Asian countries, and it shows an increasing trend in youth population who suffer from hair loss problems influenced with the raised pressures of social, working, living, and other reasons, as well as the aggravation of environmental pollutions [1].

Up to date, there are two major kinds of medicines to treat alopecia including 5*α*-reductase inhibitor represented by finasteride, and the vasodilator represented by minoxidil. These two kinds of medicines show therapeutic effects, but they also have significant adverse effects of continuing hair loss after they stop using them [2, 3].

Natural products have been providing valuable ideas for researchers to invent new drug molecules, and researchers are increasingly interested in finding and discovering therapeutic biochemical molecules from natural products. Compared with synthetic compounds, natural product molecules provide more options for the treatment of diseases, including fewer side effects, cheaper prices, and more compatibility with humans [4]. The classification of approved drug sources indicates that 6% of approved drugs are originated from natural products, while 26% of small molecule drugs are derivatives of natural products [5]. Efforts have been made to explore the use of natural products in hair care, with the goal of discovering natural active substances that prevent hair loss without adverse effects. A number of medicinal herbs were reported to have such activity, such as *Angelica sinensis* [6], *Eclipta alba* [7], and *Thuja orientalis* [8].

*Anemarrhena asphodeloides* is commonly used in the treatment of metabolic disorders in traditional Chinese medicine due to its therapeutic activities, such as antipyretic, alleviating inflammation, platelet aggregation inhibition, and antidiabetic effect [9–11]. Some defined ingredients of *A. asphodeloides* have been tested for pharmacological effects, for example, mangiferin, which helps to protect human skin keratinocyte cells against hydrogen peroxide-induced damage by scavenging intracellular reactive oxygen species, superoxide free radicals, and hydroxyl free radicals [12]; it was reported that timosaponin AIII exhibits antitumor effect [10] and timosaponin BII has protective effects against cerebral ischaemic injury [13].

The crude methanol extract of *A. asphodeloides* has estrogenic activity [14], while the diethyl ether extract shows testosterone 5*α*-reductase inhibitory activity [15]. These bioactivities suggest a potential for alleviating androgenetic alopecia. Thus, the effect of timosaponin BII obtained from *A. asphodeloides* on hair growth of C57BL/6 male mice was investigated in the present study [16].

## 2. Material and Methods

### 2.1. Materials

Timosaponin BII (Chengdu Must Bio Biotechnical Co., Ltd., China) was extracted from rhizomes of *A. asphodeloides* and purchased as a content of 98% purified by HPLC. Antibodies and reagents used in this study were as follows: anti-*β*-catenin (CST#9582, Cell Signaling Technology, USA), anti-Wnt3a (CST#2721, Cell Signaling Technology, USA), anti-Wnt10b (ab70816, Abcam, USA), hematoxylin (Beijing Zhongshan Jingqiao Biotechnical Co., Ltd., China), eosin (Shanghai Aladdin Bio-Chem Technology Co. LTD, China), minoxidil (Shanghai Aladdin Bio-Chem Technology Co. LTD, China), dimethyl sulfoxide (DMSO), and other reagents (Sigma-Aldrich, USA).

### 2.2. Experimental Animals

Male C57BL/6 mice (6-week-old, 18-20 g) purchased from Shanghai SLAC Laboratory Animal Center Inc. (Shanghai, China) were treated after acclimatizing to laboratory conditions for 1 week. Mice were fed by standard mouse food and water and stayed in an environment with a 12-hour light/dark cycle,23 ± 2°Cof temperature, and 35-60% of humidity, respectively. After one week adaptive period, 7-week-old mice were used for experiments because hair follicles of the 6- to 9-week-old C57BL/6 mice are shown to be in the telogen stage of the hair cycle [17, 18]. The anagen phase was then induced in the dorsal skin of the mice by shaving, which led to a synchronized development of anagen hair follicles. All animal procedures were performed according to the Guide for the Care and Use of Laboratory Animals of the South China University of Technology.

### 2.3. *In Vivo* Studies on Hair Growth

The mice were randomly divided into 4 groups (5 male mice each). After acclimatization for 7 days, all mice were anesthetized with an intraperitoneal injection of pentobarbital sodium (3%). The dorsal areas (approximately 2 cm in horizontal length and 4 cm in longitudinal length) of the mice were denuded with hair clippers and electrical shavers. Animals in the group of blank control received distilled water (75 *μ*L) with an equal volume of mixtures containing propylene glycol (96.5%, v/v) and ethanol (3.5%, v/v). To prepare the solution for the positive control group, minoxidil was dissolved in a mixture of propylene glycol (96.5%, v/v) and ethanol (3.5%, v/v) to a content of 4% (w/w), and then added an equal volume of distilled water to reduce the concentration of minoxidil to 2%. For the two sample groups, solutions containing timosaponin BII (0.5% and 2.5%, respectively) were prepared as described above. Equal quantities of prepared solutions (150 *μ*L) were topically applied to the denuded area of mice once a day for 15 days.

### 2.4. Skin Brightness

The skin color starts turning from white to gray-black when it converts from the telogen phase to the anagen phase [19]. As the darker and thicker hair follicles produced over time, a decreasing skin brightness of the dorsal skin may indicate the conversion of the resting hair follicles (telogen phase) to growing ones (anagen phase). The dorsal skin color was observed and measured by a chromatic meter (NH300, Shenzhen Threenh Technology Co., Ltd., China), and the *L* value of the hairless area on the 9th and 11th day were recorded and analyzed.

### 2.5. Qualitative Studies on Hair Growth

The difference in hair growth in each group was determined by visual observation and was recorded by taking photographs (Nikon D7500, Nikon Corporation, Japan). On the 11th, 14th, and 15th day, the qualitative hair growth was evaluated by analyzing the photographs with Image J software through which the percentages of the regions of interest was calculated by the equation [(black skin/total skin) × 100%], and this was done for each mouse in the 4 groups.

### 2.6. Histological Preparation

The dorsal skin of mice was isolated to examine histological features on the 15th day after depilation. Individual skin samples were fixed in 10% neutral buffered formalin at 4°C for 24 h and then washed by PBS (pH 7.4). Fixed samples were dehydrated through an ascending series of graded ethanol, cleared in xylene, and embedded in paraffin blocks [8]. Subsequently, the samples were cut either longitudinally or transversely into 4-*μ*m-thick sections with a microtome (Leica RM2235, Leica Biosystems, Germany).

### 2.7. Quantitative Histomorphometry

To quantify the hair growth-promoting activity, histomorphometric analysis was performed, and individual hair follicles were classified following Chase's protocol [20]. Sections of dorsal skin were stained with hematoxylin and eosin, and then, the histological morphology was examined using light microscopy (Eclipse 90i, Nikon Corporation, Japan). Digital photomicrographs of slides were taken at a fixed magnification of 40x. The number of hair follicles in deep subcutis was determined using the microscope.

### 2.8. Immunohistochemistry Analysis

The paraffin sections prepared above were dewaxed and then soaked into 3% H_2_O_2_ for 10 min and blocked with normal goat serum for 30 min. Then, the sections were incubated with primary antibodies against *β*-catenin (CST#9582, Cell Signaling Technology, USA), Wnt3a (CST#2721, Cell Signaling Technology, USA), or Wnt10b (ab70816, Abcam, USA) at 4°C overnight. Then, the sections were treated with an ImmunoCruz rabbit ABC Staining System (sc-2018, Santa Cruz Biotechnology, USA) according to the instructions and photographed by a microscope. The relative expression levels of *β*-catenin, Wnt3a, and Wnt10b were analyzed by the Image Pro-Plus 6.0 software. Briefly, images were converted into a black and white mode at first; then, the integrated optical density (IOD) and the area of the positive region (AREA) were calculated; finally, the mean density is obtained as IOD/AREA to indicate the relative expression levels [21].

### 2.9. Statistical Analysis

The experimental data were expressed as mean ± standard deviation. Student's *t* test was used to determine the statistical significance (*P* < 0.05) of the differences between the values for the various experimental and control groups. The software GraphPad Prism was used for the statistical analysis.

## 3. Results

### 3.1. *In Vivo* Hair Growth Effect

The hair growth of the shaved area affected by timosaponin BII was observed on days 11, 14, and 15 of the experiment; the results are shown in Figure 1. On day 11, there were few hair regrowing area in every group (Figure 1(a)), while the skin brightness was getting darker in the group of 2% minoxidil and 0.5% timosaponin BII (Figure 1(c)).

In comparison to the blank control, the hair appeared denser in the group treated with 0.5% timosaponin BII on days 14 and 15 (Figure 1(a)). However, in the group treated with 2.5% timosaponin BII, the hair looked sparse compared to the positive control (2% minoxidil). Measuring the regrowing area exhibited that group treated with 0.5% timosaponin BII showed a significant increase compared to the blank control, which is comparable to the group treated with 2% minoxidil (Figure 1(b)). On day 14, most of the mice in groups treated with minoxidil and timosaponin BII showed a rapid growth which indicated that their dorsal skin entered into the anagen phase evidently.

The C57BL/6 mouse dorsal hair has a time-synchronized hair growth cycle. The depilated mouse skin in the telogen phase is pink and darkens along with anagen initiation and then turns into gray. In this study, the hair follicles started turning darker on day 9 although no newborn hair could be observed. The skin brightness *L* value was measured, and the results are shown in Figure 1(c). The group of 0.5% timosaponin BII treatment showed the lowest *L* value on both days, indicating the fastest conversion of the hair follicles from telogen to anagen. From the data of the hair regrowing area and dorsal skin brightness test (Figure 1), 2.5% timosaponin BII treatment exhibited no remarkable effect on hair growth, indicating that an appropriate concentration is required.

### 3.2. Growth of Hair Follicle

An increase in the number and size of hair follicles has been considered as an indicator of the transition of hair growth from the telogen to anagen phases [22]. To investigate the progression of hair follicles in the hair cycle, hematoxylin-eosin staining was performed, since an increase in the size and number of hair follicles can be observed in the deep subcutis during the anagen phase [23]. The thickness of the subcutis layer increasing level and presence of the hair follicles are taken as the evidence for the transition from telogen to anagen phase during the hair follicle cycle.

In the representative longitudinal sections of day 15 dorsal skin, the number of hair follicles increased in the timosaponin BII-treated group, compared to the control group (Figure 2(a)). The horizontal sections of the day 15 dorsal skin are also shown in Figure 2(a), and the result of counting the hair follicles is shown in Figure 2(b). In the animals treated with timosaponin BII and minoxidil, the number of hair follicles was more than that of the blank control group, which indicated a clear transition from the telogen phase to the anagen phase of hair growth was induced.

### 3.3. Expression of *β*-Catenin, Wnt3a, and Wnt10b

In order to explain the underlying mechanism of the anagen phase induction in the timosaponin BII treatment group, immunohistochemistry analysis with anti-*β*-catenin and anti-Wnt antibodies was performed. It has been reported that the activation of *β*-catenin/Wnt pathway was one of the pathways that related to anagen phase induction [24]. The expression levels of *β*-catenin and Wnt10b in the timosaponin BII-treated group were higher than those in the blank control group and were comparative to the minoxidil treatment group, but there was no significant difference in the Wnt3a level (Figure 3).

## 4. Discussion

Hair loss or alopecia has increasingly become a major concern for millions of consumers worldwide. This has then raised widespread interests among cosmetologists and dermatologists. For more than 30 years, people have known that minoxidil can stimulate hair growth, but it also has obvious adverse effects, such as itching, dryness, or local irritation [25]. *Anemarrhena asphodeloides* was reported to have a wide range of effects such as 5*α*-reductase inhibition[15], anti-inflammation [12], and repairing human renal endothelial damage [26]. However, currently, there is no research on the mechanism of the hair growth-promoting activity of *A. asphodeloides*. In this study, we explored the effect of timosaponin BII extracted from *A. asphodeloides* on the activity of promoting hair growth in C57BL/6 male mice.

C57BL/6 mice are commonly used models for screening compounds that promote hair growth, because their pigmentation in the body depends on hair follicle melanocytes, which generate pigments only during the anagen phase [8]. In our study, the results showed that timosaponin BII can induce the animal hair follicle to transit from the telogen phase to the anagen phase. Compared with the control group, the 0.5% timosaponin BII treatment group had the lowest *L* value on the 9th day, and the dorsal skin started to turn darker. Since C57BL/6 mice only produce pigments in the anagen phase, the darker dorsal skin indicated an earlier transition to the anagen phase, while the control group shows a delayed transition. The hair regrowing area was measured, and the 0.5% timosaponin BII treatment group was significantly larger than the control group, which was comparative to the 2% minoxidil group. On the 15th day, the hair of all groups grew rapidly, indicating that the dorsal skin had entered the anagen phase. In addition, compared with the control, the size and shape of the hair follicles in the timosaponin BII and the minoxidil groups looked larger, rounder, and plumper, thus supporting the hair growth-promoting effects of timosaponin BII from the *A. asphodeloides*. During the entire experiment, no erythema, edema, and skin scaling/dryness were observed on any animal's application site, which suggests that there is no risk of irritation at the dose level of timosaponin BII.

It is well known that various growth factors and signal pathways are related to hair growth and hair follicle cycle [22, 27], and the Wnt/*β*-catenin pathway plays an important role in the development and growth of hair follicles and in the proliferation and regulation of embryonic as well as adult stem cell activity [28]. To reveal the molecule mechanism of the hair growth-promoting effect, the expression levels of *β*-catenin, Wnt3a, and Wnt10b were detected after receiving treatment of timosaponin BII for 15 days. The expression levels of *β*-catenin and Wnt10b in the temosaponin BII treatment group were significantly higher than those in the control group and were comparative to the minoxidil group. Interestingly, the expression level of Wnt3a remained comparable in the three groups. This may indicate that Wnt10b and *β*-catenin have a greater effect on the anagen phase of hair follicles induced by timosaponin BII, but further study is needed. In addition, detailed clinical trials and research should be conducted to determine the efficacy of timosaponin BII in the growth of alopecia patients and consumers.

In conclusion, the present study is the first to show that the timosaponin BII extracted from *A. asphodeloides* promotes hair growth by inducing the anagen phase in telogenic C57BL/6 mice. In mice treated with timosaponin BII, an increase in the number and size of hair follicles can be observed, and the regrowing area of hair is measured, which is an evidence of the induced anagen phase. Immunohistochemical analysis revealed an increase in the expression of *β*-catenin and Wnt10b. Together, these results indicate that timosaponin BII may be a potential hair growth promoter.

## Figures and Tables

**Figure 1:** Hair growth-promoting effects of timosaponin BII. The dorsal skins of 7-week-old C57BL/6 mice were shaved and topically applied with water (blank control), 2% minoxidil (positive control), 0.5% timosaponin BII, and 2.5% timosaponin BII (samples groups), respectively. (a) The back of the mice was photographed on days 11, 14, and 15. (b) The hair regrowing area. (c) Skin brightness (indicated as *L* value) of the hairless area on day 9 and day 11. The data are presented as the mean ± SD, *n* = 5, compared with the blank control group, ^∗^*P* < 0.05.

**Figure 2:** Hair follicle growth in the dorsal skins of C57BL/6 mice after topical application with minoxidil (2%) and timosaponin BII (0.5%) for 15 days. Water was used as the blank control, and sections were analyzed using hematoxylin-eosin staining. (a) Longitudinal and horizontal sections of the dorsal skins were stained, and the image shown is a representative picture of mice (green line indicates the junction of the epidermis, dermis, and subcutis). (b) Quantitative histomorphometric analysis of hair follicle number. The data are presented as the mean ± SD, *n* = 5, compared with the blank control group, ^∗^*P* < 0.05.

**Figure 3:** Immunohistochemistry analysis of *β*-catenin, Wnt3a, and Wnt10b in the dorsal skins of C57BL/6 mice after topical application with minoxidil (2%) and timosaponin BII (0.5%) for 15 days. Water was used as blank control. (a) Representative pictures of immunohistochemically stained sections of the dorsal skins. (b) The relative expression levels of proteins indicated as mean density. The data are presented as the mean ± SD, *n* = 5; compared with the blank control group, ^∗^*P* < 0.05.

## Data Availability

The raw data supporting the conclusions of this article will be made available by the corresponding author, without undue reservation, to any qualified researcher.
